# The In Vitro Antimicrobial and Antibiofilm Activities of Lysozyme against Gram-Positive Bacteria

This article has been retracted.

**DOI:** 10.1155/2022/4559982

**Published:** 2022-08-10

**Authors:** Fang Liu, Xing Wang, Lijie Huang, Xinling Wang, Lili Kong, Jinyou Duan, Xiaoli Zhang, Haibo Mu, Jianguo He

**Affiliations:** ^1^Department of Clinical Laboratory, Chongqing Red Cross Hospital, People's Hospital of Jiangbei District, Chongqing 400020, China; ^2^Shaanxi Key Laboratory of Natural Products & Chemical Biology, College of Chemistry & Pharmacy, Northwest A&F University, Yangling, 712100 Shaanxi, China; ^3^Department of Neurosurgery, Chongqing Red Cross Hospital, People's Hospital of Jiangbei District, Chongqing 400020, China

## Abstract

**Objective:**

To analyze the in vitro antibacterial and antibiofilm activities of lysozyme (LYS) and its combination with various drugs against Gram-positive bacteria (GPB, *n* = 9), thus to provide an exploration direction for drug development.

**Methods:**

The minimum inhibitory concentrations (MICs) of linezolid (LZD), amikacin (AMK), ceftriaxone/sulbactam (CRO/SBT), cefotaxime/sulbactam (CTX/SBT), piperacillin/sulbactam (PIP/SBT), doxycycline (DOX), levofloxacin (LVX), amoxicillin/clavulanate potassium (7 : 1, AK71), imipenem (IPM), azithromycin (AZM), and their combinations with LYS were determined with tuber twice dilution. The antimicrobial and antibiofilm activities of LYS, AZM, LVX, and their combinations with others were evaluated through MTT and crystal violet assay.

**Results:**

High-dose LYS (30 *μ*g/mL) combined with PIP/SBT and AK71, respectively, showed synergistic antibacterial activities against methicillin-resistant *Staphylococcus aureus* (MRSA), while it showed no synergistic activities when combined with other drugs. LYS and AZM inhibited the biofilm formation of one MRSA strain, but they and LVX had no similar activities against methicillin-resistant *Staphylococcus epidermidis* (MRSE) or vancomycin-resistant *Enterococcus faecium* (VREF). Particularly, LYS increased the permeability of biofilms of MRSA 33 and exhibited antibiofilm activities against MRSA 31 (inhibition rate = 38.1%) and MRSE 61 (inhibition rate = 46.6%). The combinations of PIP/SBT+LYS, AMK+LYS, and LZD+LYS showed stronger antibiofilm activities against MRSA 62, MRSE 62, MRSE 63, and VREF 11.

**Conclusion:**

The antimicrobial and antibiofilm activities of LYS against MRSA were better than AZM, while that of LYS against MRSE and VREF, respectively, was similar with AZM and LVX.

## 1. Introduction

Lysozyme (LYS, 1,4-*β*-N-acetylmurmidase), a single-chain alkaline protein composed of 129 amino acid residues with four pairs of disulfide bonds in the molecule, can decompose mucopolysaccharides [1]. It catalyzes the breaking of *β*-1,4-glycosidic bonds of peptidoglycan in bacterial cell walls [1, 2] and exerts broad-spectrum antibacterial activities against Gram-negative bacteria (GNB) and Gram-positive bacteria (GPB) in vitro [2]. LYS is present not only in human [3] but also in the egg whites of most avians [4]. Additionally, LYS also has many other biological properties, such as antimicrobial [2], anti-inflammatory [5], antitumor [6, 7], and antiviral [1] activities.

The stubbornness of pathogenic bacteria associated with biofilms affected the diagnosis, treatment, and prevention of most clinical infections [8, 9]. Biofilms are any microbial communities that adhere to each other on biological or nonbiological surfaces within a spontaneous extracellular polymeric substance (EPS) matrix including polysaccharides, extracellular DNA, and proteins [8, 10–13]. The biological activity of the biofilm is dominated by surface, microbes, and EPS, so it can be destroyed by removing any one of them [14, 15].

The activities of LYS on biofilms are mediated by enzymatic targeting, and it significantly condenses the hydrophobicity of bacterial biofilms [16–18]. Besides, the biofilms of *Enterococcus faecalis* and *Staphylococcus aureus* are significantly inhibited at a high concentration of LYS (25 times of MICs) [18]. Recombinant human LYS (1.0 × 10^5^ U/mL) not only inhibits the formation of *Gardnerella vaginalis* biofilms but also degrades them. Particularly, coadministration of LYS and clindamycin or metronidazole improves the efficiency of antibiotics and the degradation of *Gardnerella vaginalis* biofilms [19]. However, the low concentration of egg white LYS (5 *μ*g/mL) cannot inhibit the biofilms of *Staphylococcus aureus* isolated from raw milk and cheese and even activate the formation of a small amount (6/25, 24%) of *Staphylococcus aureus* biofilms [20].

The production and development of bacterial biofilms have significantly increased the resistance of microbes to antibiotics, which has made many existing drugs for treating microbial infections ineffective. The formation of biofilms of methicillin-resistant *Staphylococcus aureus* (MRSA), methicillin-resistant *Staphylococcus epidermidis* (MRSE), and vancomycin-resistant *Enterococcus faecium* (VREF) protects them from linezolid (LZD) [21, 22], amikacin (AMK)[23], ceftriaxone (CRO) [24, 25], cefotaxime (CTX) [25], piperacillin (PIP), doxycycline (DOX) [26], levofloxacin (LVX) [24], amoxicillin/clavulanate [8, 27, 28], imipenem (IPM) [8], and azithromycin (AZM) [28].

To provide direction for clinical application and pharmaceutical exploitation, the in vitro antimicrobial and antibiofilm activities of LYS and its combination with LZD, AMK, ceftriaxone/sulbactam (CRO/SBT), cefotaxime/sulbactam (CTX/SBT), piperacillin/sulbactam (PIP/SBT), DOX, LVX, amoxicillin/clavulanate potassium (7 : 1, AK71), IPM, and AZM against GPB in China were analyzed in this work.

## 2. Materials and Methods

### 2.1. Bacterial Isolates

All clinical isolates were collected from Chongqing Red Cross Hospital (Chongqing, China) and sent to the Northwest A&F University (Shanxi, China) to test their susceptibility (all samples in this study were processed in the laboratory environment where the ambient temperature was 20.0°C and the relative humidity was 65%). Also, all strains were reidentified by the VITEK automatic microbial analyzer (bioMerieux, France). The sensitive *Staphylococcus aureus* (ATCC 29213) was used as the quality control. This study was approved by the Medical Ethics Committee of our hospital.

### 2.2. Source of Chemicals

The LYS, LZD, AMK, CRO/SBT, CTX/SBT, PIP/SBT, DOX, LVX, AK71, IPM, and AZM were supplied by Xiangbei Welman Pharmaceutical Co., Ltd (Hunan, China). The dimethyl sulfoxide (DMSO), methanol, glacial acetic acid, and glycerol were purchased from Chengdu Chron Chemicals Co., Ltd (Sichuan, China). The crystal violet and MTT thiazolyl were, respectively, offered by Guangdong Guanghua Technology Co., Ltd (Guangdong, China) and Adamas Reagent, Ltd (Shanghai, China). The cation-adjusted Mueller-Hinton broth (CAMHB) and fluorescein isothiocyanate-dextran (FD, MW = 40 kDa), respectively, were purchased from Qingdao Haibo Biological Technology Co., Ltd (Shandong, China) and Sigma-Aldrich Trading Co., Ltd (Shanghai, China).

### 2.3. Experimental Methods

#### 2.3.1. Determination of Minimum Inhibitory Concentrations (MICs)

The MICs of clinical isolates were determined by the microbroth dilution method which was advocated by the Clinical Laboratory Standards Institute (CLSI) in M07Ed11E [29]. Taking CAMHB as solvent and control, 0.03~16 *μ*g/mL LZD, 0.25~128 *μ*g/mL AMK, 0.0625~32 *μ*g/mL CRO/SBT, 0.0625~32 *μ*g/mL CTX/SBT, 0.5~256 *μ*g/mL PIP/SBT, 0.0625~32 *μ*g/mL DOX, 0.03~16 *μ*g/mL LVX, 0.5~256 *μ*g/mL AK71, 0.03~16 *μ*g/mL IPM, and 0.25~128 *μ*g/mL AZM were configured. The concentration of CAMHB in each group was four times the maximum concentration of the drug. Immediately, 1.0 × 10^4^ CFU/mL bacterial was added to the blank group and drug group containing 100 *μ*L CAMHB or drug. After incubating at 37°C for 16~20 h, their MICs were recorded. The parallel test was performed six times. According to CLSI criteria in M100Ed30E [30], the MICs were converted into three levels: susceptible, intermediate, and resistant in the standard dosing regimen. The breakpoint of susceptibility for the main ingredient of the medicine was used when the compounds did not have a breakpoint.

#### 2.3.2. Inhibit the Formation of Biofilms

In the experimental group, 10 *μ*L 30 *μ*g/mL LYS, 10 *μ*L 16 *μ*g/mL AZM, and 10 *μ*L 2 *μ*g/mL LVX were, respectively, added to 80 *μ*L 1.0 × 10^8^ CFU/mL bacterial solution and 10 *μ*L CAMHB, while the controls consisted of 80 *μ*L 1.0 × 10^8^ CFU/mL bacterial solution and 20 *μ*L CAMHB. All were cultured at 37°C for 24 h. The number of biofilms was determined by a crystal violet assay [31]. The parallel test was performed six times.

#### 2.3.3. Destroy Mature Biofilms

100 *μ*L 1.0 × 10^8^ CFU/mL bacteria were incubated at 37°C for 24 h to form mature biofilms. Then, they were washed three times with 0.9% NaCl to take away the planktonic bacteria. 100 *μ*L 30 *μ*g/mL LYS, 16 *μ*g/mL AZM, 2 *μ*g/mL LVX, 32 *μ*g/mL PIP/SBT, 16 *μ*g/mL AMK, and 4 *μ*g/mL LZD were added in the single drug group. In combination with the medication group, 50 *μ*L 16 *μ*g/mL AK71, 16 *μ*g/mL AZM, and 2 *μ*g/mL LVX were, respectively, combined with the 50 *μ*L 32 *μ*g/mL PIP/SBT, 16 *μ*g/mL AMK, and 4 *μ*g/mL LZD. Meanwhile, the controls were composed of 100 *μ*L CAMHB. All were cultured at 37°C for 24 h. The number of active bacteria from the biofilms was determined by an MTT assay [32]. The parallel test was performed six times.

#### 2.3.4. Effect of LYS on the Permeability of GNB Mature Biofilm

100 *μ*L 1.0 × 10^8^ CFU/mL bacteria were incubated at 37°C for 24 h to form mature biofilms. Then, they were washed three times with 0.9% NaCl to take away the planktonic bacteria. 100 *μ*L 30 *μ*g/mL LYS prepared by CAMHB was added, and the biofilms were cultured at 37°C for 5 h. After the CAMHB was aspirated, FD and phosphate buffer saline (PBS) were also mixed in the biofilms. Next, the biofilms were cultured at 37°C for 20 min, washed by PBS three times, and 2 mL PBS was added. Subsequently, the biofilms were hung with a cell spatula (Fisherbrand, United States), and their fluorescence intensities were measured by a fluorescence spectrophotometer after mixing well (excitation wavelength/emission wavelength = 490 nm/520 nm). Parallel trials were conducted six times. The controls were treated with FD only and without LYS. The greater the fluorescence intensity, the more FD in the biofilms, which suggested that the permeability of the biofilm increased, resulting in a greater amount of FD entering the biofilms.

### 2.4. Statistical Analysis

All data were processed by the SPSS software and expressed as mean ± standard deviation (SD). The Satterthwaite approximate *t*-test was used for comparison between groups. ^∗^*P* < 0.05, ^∗∗^*P* < 0.01, and ^∗∗∗^*P* < 0.001 mean that the statistical difference was present, significant, and extremely significant.

## 3. Results

### 3.1. MICs Level of Various Drugs and their Combination with LYS

The MICs (*μ*g/mL) of various drugs and their combination with LYS against different species of clinical isolated GPB are shown in Table 1. For MRSA, the MICs of PIP/SBT (32 *μ*g/mL) and AK71 (16 *μ*g/mL) decreased by one or more levels when combined with high-dose LYS (30 *μ*g/mL), suggesting that these two combinations showed a synergistic antibacterial effect. However, LZD, AMK, CRO/SBT, CTX/SBT, DOX, LVX, IPM, and AZM, respectively, combined with LYS (10 or 30 *μ*g/mL) had no synergistic antimicrobial activities against MRSA, MRSE, and VREF.

### 3.2. Inhibit the Formation of Biofilms

The activities of LYS and AZM on the formation of GPB biofilm assessed by crystal violet stain are displayed in Table 2. The OD values of LYS against MRSA 31 (78.4%, *P* < 0.05), MRSE (75.6%, *P* > 0.05; 71.5%, *P* > 0.05; and 87.3%, *P* > 0.05), VREF 11 (97.0%, *P* > 0.05), VREF 13 (93.3%, *P* > 0.05), and AZM against MRSA 31 (73.2%, *P* < 0.05) were larger than the control with a percentage < 100%, while only LYS against MRSA 31 and AZM against MRSA 31 showed a statistical difference to the control (*P* < 0.05). Both LYS and AZM significantly inhibited the biofilm formation of MRSA 31, but they did not show any significant effects on MRSE and VREF.

### 3.3. Destroy Mature Biofilms

#### 3.3.1. MRSA

The effect of LYS on the permeability of MRSA mature biofilms is illustrated in Figure 1. LYS treatment induced a stronger fluorescence intensity of MRSA 33 biofilm than FD alone (*P* = 0.0381), indicating that LYS (30 *μ*g/mL) was able to increase the permeability of MRSA 33 biofilm. Additionally, the viable bacteria in the mature biofilm of MRSA detected by MTT after treatment with LYS, AZM, and their combinations with PIP/SBT are demonstrated in Table 3. The OD values of LYS against MRSA 31 (61.9%, *P* < 0.05), AZM against MRSA 62 (98.7%, *P* >0.05), PIP/SBT against MRSA 31 (95.9%, *P* > 0.05) and MRSA 33 (93.0%, *P* > 0.05), PIP/SBT+LYS against MRSA (64.6%, *P* < 0.05; 62.9%, *P* > 0.05; and 91.8%, *P* >0.05), and PIP/SBT+AZM against MRSA (90.6%, *P* > 0.05; 74.3%, *P* > 0.05; and 66.4%, *P* > 0.05) were smaller than the control with percentages < 100%, while only the values of LYS against MRSA 31 and PIP/SBT+LYS against MRSA 31 showed significant difference (*P* < 0.05). Therefore, LYS alone had antibacterial activity against MRSA 31 in mature biofilm, but AZM did not show this effect. Moreover, the percentage of OD value about PIP/SBT+LYS against MRSA 62 was less than 100% and was obviously associated with that of LYS (83.5%, *P* < 0.01), suggesting that the combination of PIP/SBT and LYS increased the antimicrobial activity of PIP/SBT against MRSA 62 in biofilm. Similarly, the combination of LYS and PIP/SBT also improved the antibacterial activity of LYS against MRSA 33 and MRSA 62, resulting from the OD value of PIP/SBT+LYS against MRSA 33 and MRSA 62 being significantly related to that of PIP/SBT (53.0%, *P* < 0.05; 93.0%, *P* < 0.01). Meanwhile, the OD values of PIP/SBT+AZM were visibly associated with that of AZM against MRSA 33 and MRSA 62 (63.4%, *P* < 0.05; 60.4%, *P* < 0.05) and PIP/SBT against MRSA 33 (80.0%, *P* < 0.01), respectively, indicating that the combination of PIP/SBT and AZM strengthened the antimicrobial activities of PIP/SBT against MRSA 33, MRSA 62, and AZM against MRSA 33 in biofilms.

#### 3.3.2. MRSE

The viable bacteria in the mature biofilm of MRSE detected by MTT after treatment with LYS, AZM, and their combinations with AMK are shown in Table 4. The OD values of LYS (53.4%, *P* < 0.05; 71.8%, *P* > 0.05; and 76.1%, *P* >0.05), AZM (86.1%, *P* > 0.05; 74.7%, *P* > 0.05; and 49.2%, *P* < 0.05), AMK (21.7%, *P* < 0.05; 80.7%, *P* > 0.05; and 30.4%, *P* < 0.01), AMK+LYS (16.1%, *P* < 0.05; 44.5%, *P* < 0.05; and 13.3%, *P* < 0.01), and AMK+AZM (16.3%, *P* < 0.05; 38.5%, *P* < 0.05; and 15.0%, *P* < 0.01) against MRSE were less than the control with percentages < 100%, but only the values of LYS against MRSE 61, AZM against MRSE 63, AMK against MRSE 61 and MRSE 63, AMK+LYS against MRSE, and AMK+AZM against MRSE displayed a statistical difference (*P* < 0.05). Thus, LYS behaved with bactericidal activity against MRSE 61 in biofilms, which was consistent with the situation of AZM against MRSE 63 and AMK against MRSE 61 and MRSE 63. Furthermore, the OD values of AMK+LYS were significantly associated with that of LYS against MRSE (31.2%, *P* < 0.05; 62.0%, *P* < 0.05; and 17.5%, *P* < 0.05) and AMK against MRSE 62 (59.6%, *P* < 0.05) and MRSE 63 (27.1%, *P* < 0.05), suggesting that the combination of LYS and AMK heightened the antimicrobial activity of LYS against MRSE and AMK against MRSE 62 and MRSE 63 in biofilms. The combination of AZM and AMK raised the antibacterial activity of AMK against MRSE and AZM against MRSE 62 and MRSE 63 in biofilms because the OD values of AMK+AZM were obviously related to that of AZM against MRSE (30.6%, *P* < 0.05; 53.6%, *P* < 0.05; and 19.7%, *P* < 0.01) and AMK against MRSE 62 (47.7%, *P* < 0.001) and MRSE 63 (49.4%, *P* < 0.05).

#### 3.3.3. VREF

The viable bacteria in the mature biofilm of VREF detected by MTT after treatment with LYS, LVX, and their combinations with LZD are displayed in Table 5. The OD values of LYS against VREF 12 (98.3%, *P* > 0.05), VREF 13 (91.5%, *P* > 0.05), LVX against VREF 12 (93.8%, *P* > 0.05) and VREF 13 (87.3%, *P* > 0.05), LZD against VREF (61.7%, *P* < 0.05; 55.1%, *P* < 0.01; and 78.9%, *P* > 0.05), LZD+LYS against VREF (79.3%, *P* > 0.05; 61.2%, *P* > 0.05; and 78.9%, *P* > 0.05), and LZD+LVX against VREF (69.7%, *P* < 0.05; 53.4%, *P* < 0.05; and 74.6%, *P* > 0.05) were lower than the controls, while only the values of LZD against VREF 11 and VREF 12 and LZD+LVX against VREF 11 and VREF 12 were notable (*P* < 0.05). What is more, the value of LZD+LYS against VREF 11 was significantly associated with that of LYS (70.3%, *P* < 0.05), implying that the combination of LZD and LYS improved the antimicrobial activity of LZD against VREF 11 in biofilms. The OD values of LZD+LVX against VREF 11 (61.8%, *P* < 0.01) and VREF 12 (54.3%, *P* < 0.01) were obviously related to that of LVX, so the combination of LZD and LVX enhanced the antibacterial activity of LZD against VREF 11 and VREF 12 in biofilms.

## 4. Discussion

The concentration of various drugs in the antibiofilm activity test was selected based on their breakpoint of susceptibility in CLSI criteria [30]. The concentration of LYS, AZM, PIP/SBT, AMK, LVX, and LZD in assessing their antimicrobial and antibiofilm activities against MRSA, MRSE, and VREF, respectively, was 30, 16, 32, 16, 2, and 4 *μ*g/mL. Moreover, when high-dose LYS (30 *μ*g/mL) was used in combination with PIP/SBT and AK71, they produced synergistic antibacterial effects against MRSA, MRSE, and VREF. When LYS was used in combination with LZD, AMK, CRO/SBT, CTX/SBT, DOX, LVX, IPM, and AZM, there was neither obvious synergy nor antagonism against MRSA, MRSE, and VREF. Therefore, LYS might be a potential and safe antibacterial adjuvant medication against GPB, especially when it was used in combination with PIP/SBT and AK71.

Biofilms made it difficult for conventional antibiotics to penetrate into bacterial cells and enhanced the resistance of microbes [33, 34]. The process by which bacteria form biofilms included adhesion to the biological or nonbiological surfaces, development of structure, maturation, and diffusion from the biofilms to return to a planktonic state [14, 15, 34]. Except for LYS and AZM against MRSA 31, LYS, AZM, and LVX were unable to inhibit the formation of MRSA, MRSE, and VREF biofilms. Consequently, LYS and LVX showed no activities against the adhesion and structural development of most MRSA and MRSE. Similarly, LYS and LVX did not affect the adhesion and structural development of VREF.

Additionally, high-dose LYS (30 *μ*g/mL) not only killed the MRSA 33 in biofilms but also increased the permeability of the biofilms of MRSA 31 and ultimately eliminated bacteria in biofilms. In the same way, LYS had antibacterial activities against MRSE 62 and MRSE 63 in biofilms. Thence, LYS might exhibit its antibiofilm activities against MRSA and MRSE by destroying the permeability of mature bacterial biofilms or preventing the microbes in the biofilms from returning to their planktonic state. Moreover, the combination of PIP/SBT+LYS, AMK+LYS, and LZD+LYS, respectively, increased the antimicrobial activity of PIP/SBT against MRSA 62, AMK against MRSE 62 and MRSE 63, and LZD against VREF 11 in biofilms. Most importantly, the biofilms of MRSA were one of the main causes of eye infections related to contact lenses [35], bloodstream infections, and urinary tract infections associated with catheters [8, 36], so LYS might be a potential treatment for these three types of infections, and the combination of PIP/SBT+LYS was more effective than LYS. The biofilms of VREF played an important role in canine periodontal disease [37], resulting in the combination of LZD+LYS that might be efficacious in relieving the symptoms of this disease. *Staphylococcus epidermidis*, a coagulase-negative staphylococcus (CoNS), lacked aggressive virulence factors, and their pathogenicity was attributed to their ability to form biofilms [38]. It also accounted for approximately 70% of all CoNS in human skin and was the foremost cause of severe bloodstream infections and one of the most common causes of healthcare-related infections [38–40]. Hence, the combination of LYS and LZD was a possible option to alleviate the severe bloodstream infections and healthcare-related infections caused by MRSE.

However, due to the small number of clinical isolates studied in this work, it was not yet possible to accurately describe the antibiofilm activities of LYS and its combination with various drugs against GNB. Research on large samples still needed to be carried out to provide directions for screening suitable antibiofilm drugs.

## 5. Conclusion

The combinations of PIP/SBT and high-dose LYS (30 *μ*g/mL), AK71, and high-dose LYS showed a synergistic antibacterial activity for their MICs that were lower than that used alone by one or more levels, while LZD, AMK, CRO/SBT, CTX/SBT, DOX, LVX, IPM, and AZM, respectively, combined with LYS did not display the similar activities against MRSA, MRSE, and VREF. Besides, both LYS and AZM significantly inhibited the formation of biofilm in one of the three MRSA strains, but they were unable to inhibit the biofilm formation of each of the three MRSE or VREF isolates. Particularly, high-dose LYS obviously increased the permeability of the biofilms of one of the three MRSA strains (MRSA 33). Moreover, LYS used alone had antibacterial activity against MRSA 31, and the combination of PIP/SBT+LYS increased the antimicrobial activity of PIP/SBT against MRSA 62 in biofilms, but AZM did not show such effect. Besides, LYS behaved with bactericidal activity against MRSE 61, and the combination of AMK+LYS heightened the antimicrobial activity of AMK against MRSE 62 and MRSE 63 in biofilms. AZM shows antibacterial activity against MRSE 63, and the combination of AMK+AZM raised the antibacterial activity of AMK against three MRSE isolates in biofilms. LYS did not have antibacterial activity against VREF when used alone, while the combination of LZD+LYS improved the antimicrobial activity of LZD against VREF 11 in biofilms. Also, LVX could not inhibit VREF, and the combination of LZD+LVX enhanced the antibacterial activity of LZD against VREF 11 and VREF 12 in biofilms. In short, the antimicrobial and antibiofilm activities of LYS against MRSA were better than AZM, while that of LYS against MRSE and VREF, respectively, was similar to AZM and LVX.

## Figures and Tables

**Figure 1:** Effect of LYS on the permeability of MESA mature biofilms. MRSA 31, MRSA 33, and MRSA 62 represented three different clinical isolates. MRSA: methicillin-resistant *Staphylococcus aureus*; RM, LYS: lysozyme, 30 *μ*g/mL; FD: fluorescein isothiocyanate-dextran, MW = 40 kDa. ^∗^*P* < 0.05, ^∗∗^*P* < 0.01, and ^∗∗∗^*P* < 0.001 compared with the control.

**Table 1:** The MICs (*μ*g/mL) of various drugs and their combination with LYS against different species of clinical isolated GPB.

No.	Drugs	Isolates		Use alone	Combinations	
					+10 *μ*g/mL LYS	+30 *μ*g/mL LYS
1	LZD	MRSA	31 ^a^	1	1	1
			33	1	1	1
			62	1	1	1
		MRSE	61	1	1	1
			62	1	1	1
			63	1	1	1
		VREF	11	2	2	1
			12	1	1	1
			13	1	1	1
2	AMK	MRSA	31	1	1	1
			33	2	1	4
			62	2	4	4
		MRSE	61	<0.5	<0.5	<0.5
			62	2	2	2
			63	2	2	2
		VREF	11	>256	>256	>256
			12	>256	>256	>256
			13	>256	>256	>256
3	CRO/SBT	MRSA	31	>256	>256	>256
			33	32	32	16
			62	8	8	8
		MRSE	61	>32	>32	>32
			62	4	8	8
			63	16	16	32
		VREF	11	>256	>256	>256
			12	>32	>32	>32
			13	>32	>32	>32
4	CTX/SBT	MRSA	31	>256	>256	>256
			33	16	16	8
			62	8	8	8
		MRSE	61	>32	>32	>32
			62	>32	>32	>32
			63	8	8	4
		VREF	11	>256	>256	>256
			12	>32	>32	>32
			13	>32	>32	>32
5	PIP/SBT	MRSA	31	256	256	128
			33	16	16	8
			62	8	8	4
		MRSE	61	128	128	64
			62	32	32	16
			63	2	2	2
		VREF	11	>256	>256	>256
			12	>256	>256	>256
			13	>256	>256	>256
6	DOX	MRSA	31	0.5	0.5	0.5
			33	<0.0625	<0.0625	<0.0625
			62	2	2	2
		MRSE	61	<0.0625	<0.0625	<0.0625
			62	<0.0625	<0.0625	<0.0625
			63	1	1	1
		VREF	11	<0.0625	<0.0625	<0.0625
			12	8	8	4
			13	<0.0625	0.125	<0.0625
7	LVX	MRSA	31	8	8	8
			33	0.25	0.25	0.25
			62	0.5	0.5	0.5
		MRSE	61	16	16	8
			62	2	2	2
			63	8	8	8
		VREF	11	32	32	32
			12	>16	>16	>16
			13	>16	>16	>16
8	AK71	MRSA	31	64	64	32
			33	8	4	2
			62	2	4	<0.5
		MRSE	61	32	16	8
			62	<0.5	<0.5	<0.5
			63	1	<0.5	1
		VREF	11	>256	>256	>256
			12	128	128	128
			13	>256	>256	>256
9	IPM	MRSA	31	64	64	64
			33	0.5	0.5	0.5
			62	<0.125	<0.125	<0.125
		MRSE	61	16	2	0.5
			62	0.125	0.25	0.25
			63	1	1	1
		VREF	11	>256	>256	>256
			12	>32	>32	>32
			13	>32	>32	>32
10	AZM	MRSA	31	128	128	64
			33	>128	>128	>128
			62	>128	>128	>128
		MRSE	61	>128	>128	>128
			62	>128	>128	>128
			63	>128	>128	>128
		VREF	11	1	1	1
			12	>256	>256	>256
			13	>128	>128	>128

A number indicated the name of clinical isolates. MICs: minimum inhibitory concentrations; GPB: Gram-positive bacteria; MRSA: methicillin-resistant *Staphylococcus aureus*; MRSE: methicillin-resistant *Staphylococcus epidermidis*; VREF: vancomycin-resistant *Enterococcus faecium*; LYS: lysozyme; LZD: linezolid; AMK: amikacin; CRO/SBT: ceftriaxone/sulbactam; CTX/SBT: cefotaxime/sulbactam; PIP/SBT: piperacillin/sulbactam; DOX: doxycycline; LVX: levofloxacin; AK71: amoxicillin/clavulanate potassium 7 : 1; IPM: imipenem; AZM: azithromycin; –: not tested.

**Table 2:** The activities of LYS and AZM on the formation of GPB biofilms assessed by crystal violet stain.

Species	Isolates (*n* = 3)	Control		LYS		AZM	
		Values	Percentage (%)	Values	Percentage (%)	Values	Percentage (%)
MRSA	31 ^a^	0.735 ± 0.0529	100.0	0.576 ± 0.0244	78.4∗	0.538 ± 0.0360	73.2∗
	33	0.378 ± 0.0424	100.0	0.392 ± 0.0244	103.7	0.412 ± 0.0331	109.0
	62	0.243 ± 0.0264	100.0	0.270 ± 0.0244	111.1	0.259 ± 0.0200	106.6
MRSE	61	0.639 ± 0.0934	100.0	0.483 ± 0.1134	75.6	0.656 ± 0.0750	102.7
	62	0.235 ± 0.0297	100.0	0.168 ± 0.0102	71.5	0.241 ± 0.0877	102.6
	63	0.173 ± 0.0328	100.0	0.151 ± 0.0115	87.3	0.154 ± 0.0146	89.0
VREF	11	0.264 ± 0.0514	100,0	0.256 ± 0.0377	97.0	0.265 ± 0.0435	100.4
	12	0.178 ± 0.0245	100.0	0.204 ± 0.0316	114.6	0.208 ± 0.0214	116.9
	13	0.164 ± 0.0187	100.0	0.153 ± 0.0126	93.3	0.181 ± 0.0158	110.4

A number indicated the name of clinical isolates. The values of OD are shown in mean ± standard deviation (SD). The percentage was defined as (OD value of the treatment group/OD value of the control) × 100%. The concentration of LYS and AZM, respectively, was 30 and 16 *μ*g/mL. ^∗^*P* < 0.05, ^∗∗^*P* < 0.01, and ^∗∗∗^*P* < 0.001 compared with the control. GPB: Gram-positive bacteria; MRSA: methicillin-resistant *Staphylococcus aureus*; MRSE: methicillin-resistant *Staphylococcus epidermidis*; VREF: vancomycin-resistant *Enterococcus faecium*; LYS: lysozyme; AZM: azithromycin; OD: optical density.

**Table 3:** The OD of LYS, AZM, and their combinations with PIP/SBT on the mature biofilms of MRSA.

Groups	MRSA 31		MRSA 33		MRSA 62	
	Values	Percentage (%)	Values	Percentage (%)	Values	Percentage (%)
Control	0.658 ± 0.0877	100.0	0.499 ± 0.0927	100.0	0.685 ± 0.0843	100.0
LYS	0.407 ± 0.0183	61.9^∗^	0.585 ± 0.0640	117.2	0.753 ± 0.0959	109.9
AZM	0.749 ± 0.0400	113.8	0.592 ± 0.0755	118.6	0.676 ± 0.0447	98.7
PIP/SBT	0.631 ± 0.0490	95.9	0.464 ± 0.0245	93.0	0.753 ± 0.0608	109.9
A: PIP/SBT+LYS	0.425 ± 0.0217	64.6^∗^	0.314 ± 0.0212	62.9	0.629 ± 0.0436	91.8
B: PIP/SBT+AZM	0.596 ± 0.0742	90.6	0.371 ± 0.0390	74.3	0.455 ± 0.0938	66.4
Comparison between different groups						
A1: A and LYS	—	104.4	—	53.7	—	83.5^∗∗^
B1: B and AZM	—	146.4	—	63.4^∗^	—	60.4^∗^
A2: A and PIP/SBT	—	56.7	—	53.0^∗^	—	93.0^∗∗^
B2: B and PIP/SBT	—	94.5	—	80.0^∗∗^	—	60.4

The values of OD are shown in mean ± standard deviation (SD). The percentage was defined as (OD value of the treatment group/OD value of the control) × 100%. MRSA 31, MRSA 33, and MRSA 62 represented three different clinical isolates. ^∗^*P* < 0.05, ^∗∗^*P* < 0.01, and ^∗∗∗^*P* < 0.001 compared with the control. MRSA: methicillin-resistant *Staphylococcus aureus*; OD: optical density; MTT: methylthiazolyldiphenyl-tetrazolium bromide; LYS: lysozyme; AZM: azithromycin; PIP/SBT: piperacillin/sulbactam; –: not tested.

**Table 4:** The OD of LYS, AZM, and their combinations with AMK on the mature biofilms of MRSE.

Groups	MRSE 61		MRSE 62		MRSE 63	
	Values	Percentage (%)	Values	Percentage (%)	Values	Percentage (%)
Control	0.631 ± 0.0724	100.0	0.348 ± 0.0497	100.0	0.832 ± 0.1173	100.0
LYS	0.337 ± 0.0705	53.4^∗^	0.250 ± 0.0188	71.8	0.633 ± 0.0921	76.1
AZM	0.543 ± 0.0472	86.1	0.260 ± 0.0305	74.7	0.409 ± 0.0703	49.2^∗^
AMK	0.137 ± 0.0232	21.7^∗^	0.281 ± 0.01400	80.7	0.253 ± 0.02230	30.4^∗∗^
A: AMK+LYS	0.105 ± 0.0168	16.6^∗^	0.155 ± 0.01004	44.5^∗^	0.111 ± 0.0124	13.3^∗∗^
B: AMK+AZM	0.103 ± 0.0135	16.3^∗^	0.134 ± 0.0078	38.5^∗^	0.125 ± 0.0368	15.0^∗∗^
Comparison between different groups						
A1: A and LYS	—	31.2^∗^	—	62.0^∗^	—	17.5^∗^
B1: B and AZM	—	30.6^∗^	—	53.6^∗^	—	19.7^∗∗^
A2: A and AMK	—	19.3	—	59.6^∗^	—	27.1^∗∗^
B2: B and AMK	—	75.2	—	47.7^∗∗∗^	—	49.4^∗^

The values of OD are shown in mean ± standard deviation (SD). The percentage was defined as (OD value of the treatment group/OD value of the control) × 100%. MRSE 61, MRSE 62, and MRSE 63 represented three different clinical isolates. ^∗^*P* < 0.05, ^∗∗^*P* < 0.01, and ^∗∗∗^*P* < 0.001 compared with the control. MRSE: methicillin-resistant *Staphylococcus epidermidis*; OD: optical density; MTT: methylthiazolyldiphenyl-tetrazolium bromide; LYS: lysozyme; AZM: azithromycin; AMK: amikacin; –: not tested.

**Table 5:** The OD of LYS, LVX, and their combinations with LZD on the mature biofilms of VREF.

Groups	VREF 11		VREF 12		VREF 13	
	Values	Percentage (%)	Values	Percentage (%)	Values	Percentage (%)
Control	0.188 ± 0.0229	100.0	0.178 ± 0.0189	100.0	0.142 ± 0.0233	100.0
LYS	0.212 ± 0.0194	112.8	0.175 ± 0.0210	98.3	0.130 ± 0.0237	91.5
LVX	0.197 ± 0.0166	104.8	0.167 ± 0.0133	93.8	0.124 ± 0.0229	87.3
LZD	0.116 ± 0.0239	61.7^∗^	0.098 ± 0.0106	55.1^∗∗^	0.112 ± 0.0252	78.9
A: LZD+LYS	0.149 ± 0.0224	79.3	0.109 ± 0.0359	61.2	0.112 ± 0.0242	78.9
B: LZD+LVX	0.131 ± 0.0168	69.7^∗^	0.095 ± 0.0073	53.4^∗∗^	0.106 ± 0.0184	74.6
Comparison between different groups						
A1: A and LYS	—	70.3^∗^	—	62.3	—	86.2
B1: B and LVX	—	61.8^∗∗^	—	54.3^∗∗^	—	81.5
A2: A and LZD	—	75.6	—	65.3	—	90.3
B2: B and LZD	—	112.9	—	96.9	—	94.6

The values of OD are shown in mean ± standard deviation (SD). The percentage was defined as (OD value of the treatment group/OD value of the control) × 100%. VREF 11, VREF 12, and VREF 13 represented three different clinical isolates. ^∗^*P* < 0.05, ^∗∗^*P* < 0.01, and ^∗∗∗^*P* < 0.001 compared with the control. VREF: vancomycin-resistant *Enterococcus faecium*; OD: optical density; MTT: methylthiazolyldiphenyl-tetrazolium bromide; LYS: lysozyme; LVX: levofloxacin; LZD: linezolid; –: not tested.

## Data Availability

The data used to support the findings of this study are available from the corresponding authors upon request.
